The article "A Multiplexed Microfluidic PCR Assay for Sensitive and Specific Point-of-Care Detection of Chlamydia trachomatis" was published in 2012. Journal: PLoS One.

# A Multiplexed Microfluidic PCR Assay for Sensitive and Specific Point-of-Care Detection of *Chlamydia trachomatis*

**DOI:** 10.1371/journal.pone.0051685

**Published:** 2012-12-14

**Authors:** Deborah Dean, Rosemary S. Turingan, Hans-Ulrich Thomann, Anna Zolotova, James Rothschild, Sandeep J. Joseph, Timothy D. Read, Eugene Tan, Richard F. Selden

**Affiliations:** 1 Center for Immunobiology and Vaccine Development, Children’s Hospital Oakland Research Institute, Oakland, California, United States of America; 2 University of California at Berkeley and University of California at San Francisco Joint Graduate Program in Bioengineering, Berkeley, California, United States of America; 3 NetBio, Waltham, Massachusetts, United States of America; 4 Department of Medicine, Division of Infectious Diseases and Department of Human Genetics, Emory University School of Medicine, Atlanta, Georgia, United States of America; University of California Merced, United States of America

## Abstract

**Background:**

*Chlamydia trachomatis (Ct*) is the most common cause of bacterial sexually transmitted diseases (STD) worldwide. While commercial nucleic acid amplification tests (NAAT) are available for *Ct*, none are rapid or inexpensive enough to be used at the point-of-care (POC). Towards the first *Ct* POC NAAT, we developed a microfluidic assay that simultaneously interrogates nine *Ct* loci in 20 minutes.

**Methodology and Principal Findings:**

Endocervical samples were selected from 263 women at high risk for *Ct* STDs (∼35% prevalence). A head-to-head comparison was performed with the Roche-Amplicor NAAT. 129 (49.0%) and 88 (33.5%) samples were positive by multiplex and Amplicor assays, respectively. Sequencing resolved 71 discrepant samples, confirming 53 of 53 positive multiplex samples and 12 of 18 positive Amplicor samples. The sensitivity and specificity were 91.5% and 100%, and 62.4% and 95.9%, respectively, for multiplex and Amplicor assays. Positive and negative predictive values were 100% and 91%, and 94.1% and 68.6%, respectively.

**Conclusions:**

This is the first rapid multiplex approach to *Ct* detection, and the assay was also found to be superior to a commercial NAAT. In effect, nine simultaneous reactions significantly increased sensitivity and specificity. Our assay can potentially increase *Ct* detection in globally diverse clinical settings at the POC.

## Introduction

*Chlamydia trachomatis* (*Ct*) is an obligate intracellular pathogen that is responsible for the highest incidence of bacterial sexually transmitted diseases (STD) in the world today. Over 100 million cases occur each year according to the World Health Organization. The estimated cost of the approximate one million annual cases in the United States is $2.4 billion [1]. Because most infections in men and women are asymptomatic, the opportunity for unchecked transmission is high even in countries with advanced public health care systems. While antibiotics are effective in treating most uncomplicated infections to prevent the sequelae of pelvic inflammatory disease, infertility and life-threatening ectopic pregnancy, the lack of cost effective screening tests has greatly hindered infection control [2]–[4]. Furthermore, even if screening is performed, patients at high risk for STDs are less likely to return for test results [5].

The article "A Multiplexed Microfluidic PCR Assay for Sensitive and Specific Point-of-Care Detection of Chlamydia trachomatis" was published in 2012. Journal: PLoS One.

The most common tests for *Ct* screening are nucleic acid amplification tests (NAAT). They are only available in specialized clinical laboratories, and results take a day or longer to report. Although NAATs are thought to have good sensitivity and specificity, the ranges are 80–97% and 91–99%, respectively [6], [7], with a general lack of concordant results for the same sample type using different NAATs [8]–[10]. Additionally, the tests are based on interrogation of one or two loci, a limitation that can lead to false negatives. This has recently been shown for two NAATs that missed detection of a new Swedish *Ct* strain variant containing a deletion at the primer binding sites [11].

Available rapid tests have sensitivities as low as 12% and up to 95% and specificities of 97.9–100%, depending on the sample, compared with NAAT or in-house PCR tests [12]–[18]. In April 2011, CDC reiterated their recommendation for increasing *Ct* screening coverage and endorsed expedited partner therapy [19]. CDC prefers NA-based methods for *Ct* diagnosis but a 2009 CDC-led Expert Consultation Panel concluded that existing point-of-care (POC) diagnostics were unsuitable for routine use and “development of improved POC tests desirable” [20]. This need is further evidenced by a recent report of the “alarming” performance of three *Ct* POC assays with sensitivities of only 12–27% [21]. Thus, there remains a tremendous need for a sensitive, rapid, and cost effective diagnostic that is available at the POC to screen at risk populations and inform timely treatment decisions.

We developed a microfluidics-based multiplexed assay for the detection of *Ct* that can be adapted to the POC. The system simultaneously interrogates nine *Ct* loci in a 20-minute amplification reaction, and provides data in approximately one hour from sample collection, faster than any extant *Ct* NAAT. The assay is based on microfluidic modules that purify DNA from clinical samples, performs highly multiplexed amplification, and separates the amplicons electrophoretically with laser-induced fluorescence detection. Here, we evaluated the microfluidic amplification, separation and detection modules for detection of *Ct* in endocervical swabs obtained from women attending STD clinics.

The article "A Multiplexed Microfluidic PCR Assay for Sensitive and Specific Point-of-Care Detection of Chlamydia trachomatis" was published in 2012. Journal: PLoS One.

## Methods

### Study Population and Sample Collection

To ensure high rates of *Ct*, we selected endocervical swabs obtained from 15 to 24 year old females sequentially seen at STD clinics in the San Francisco Bay Area who had a history of unprotected intercourse, multiple sex partners, prior STDs, and no use of antibiotics within the previous three weeks who were not menstruating. The prevalence of *Ct* among this population is 15–19% for all comers and ∼35% for high-risk females using commercial NAATs. One swab per patient was collected using Dacron swabs and M4 media (REMEL, Lenexa, KS). Because the remnant samples were supplied to us de-identified with no trace back to patient names, the study was considered not human subjects research according to NIH and CHORI IRB guidelines.

### Sample Testing Using the Commercial Amplicor NAAT

The Roche Amplicor NAAT (Roche Diagnostics, Indianapolis, IN) amplifies a segment of the cryptic plasmid. Roche reports sensitivity and specificity of 86.5–98.9% and 91.9–98.6%, respectively. The assay does not detect the Swedish variant, although the recently released Roche cobas® 4800 CT/GC test, which reports a sensitivity of 93.8% and specificity of 100% for swabs [22], detects the variant and *omp*A. Samples were processed as recommended by the manufacturer. The Amplicor Internal Control (IC) Detection Kit was run in parallel to detect any inhibition of amplification.

### DNA Purification for the Multiplex Assay

DNA purification was performed essentially as described [23]. Briefly, 735 µl of guanidinium-proteinase K-based lysis solution was added to each tube containing the clinical swab followed by vortexing. 735 µl of absolute ethanol was added, and lysate was passed through a spin column with silica DNA-binding membrane, washed 4 times, and eluted in 30 µl Tris-EDTA (pH 8.0).

### PCR Primer Design

*Ct* amplification targets included a Multi-Locus Sequence Typing (MLST) set (*gly*A, *mdh*C, *pyk*F, *yhb*G, *lys*S, *pdh*A and *leu*S) [24], *omp*A, and the cryptic plasmid. Published whole genome sequence data of 20 *Ct* strains, representing serovars L_2_, L_2_b, A, B, D, D(s), E, F, G, and J, were utilized to locate conserved regions amenable to the design of *Ct* specific primers. Finished and whole genome shotgun sequences were searched via blastn using reference sequences from LGV strain L_2_/434/Bu. Partial sequence data from additional strains were also included. Retrieved sequences were aligned by ClustalX 2.1 [25], and primers were designed by Visual OMP Vs. 7.4.0.0. (DNA Software, Ann Arbor, MI). Finally, primers were checked for specificity by blastn against genome data including human, yeast, and other *Chlamydia* and *Chlamydophyla* species.

The article "A Multiplexed Microfluidic PCR Assay for Sensitive and Specific Point-of-Care Detection of Chlamydia trachomatis" was published in 2012. Journal: PLoS One.

Primers were designed such that amplicons were separately distinguished either by size or fluorescent label. Labels were placed at the 3′end of the forward primer. Primer pairs with high amplification signals at 50 *Ct* genome copies were chosen for use in the multiplex assembly. Primers were redesigned when primer interference (e.g., one or more amplification products disappeared on addition of new primer to the mix) was observed. Table 1 includes primers utilized for the 9-plex amplification.

**Table 1:** Selected targets, primer sequences, amplicon size, and fluorescent labels used.

Target/Primer	Locus/Gene	Label*	Amplicon [bp]	Forward (5′ to 3′)	Reverse (5′ to 3′)
*omp*A–F2/R2	*omp*A	FAM	220	GAAAAAACTCTTGAAATCGGTATTAGT	CAAAACRCGGTCGAAAACAAAG
pCT8–F/R	pCT-ORF8	FAM	349	TAGGCGTTTGTACTCCGTCACA	TTGGTTGATCGCCCAGACAATG
*pdh*A–F4/R2	*pdh*A	FAM	417	GCGGAGAAGAGGCCTATTTAGAA	GGGAGTGAAGCGCTACAAAA
*yhb*G–F4/R3	*yhb*G	TAMRA	446	CGTCCTGAYTCTGGAAAAATTCTG	ATAGATAAGAGTTCTTTTGCGTTATG
*mdh*C–F3/R2	*mdh*C	TAMRA	480	CGATCTGCGTATCTACGATATTC	GTAAAATCAGGCACTTGTTTGGC
*gly*A–F4/R4	*gly*A	ROX	450	GCCAAGAGGTGGATTGGTT	ACGATAATATTCGCAACTTCTTCC
*pyk*F–F4/R2	*pyk*F	ROX	467	AGTTTTGGAAAGCTTTGGTCG	CAAGATAAGGAGAAACTTTGAGAGC
*lys*S–F6/R6	*lys*S	ROX	497	GATGTAATGAAATGTGTGGAAAACC	TTACGCATTTGCTCTTCCAACA
*leu*S–F3/R2	*leu*S	ROX	508	AAGAAACACAAAGTAAAAGCGAAAGA	TCTGGTCGATAATCTTGAATTTCCG

* Fluorescent labels were placed at the 5′end of the forward primer.

### Microfluidic Multiplex PCR Amplification

The microfluidic biochip and rapid thermal cycler have been utilized for both forensic application and biothreat detection [23], [26]. For *Ct* detection, a 7 µl reaction mixture was amplified in 20 minutes using a 33-cycle protocol as previously described [26]. Typically, 20 ng of purified DNA was input into the amplification reaction. Amplicons were microfluidically separated and detected by laser-induced fluorescence using the Genebench-FX instrument and accompanying biochip [26].

**Figure 1:** Representative 9-plex *Ct* PCR panel with 50 genome equivalents of *C. trachomatis* (from strain H/UW-43/Cx) (A). Other *Ct* DNAs used were E/Bour, D/UW-3/Cx, G/UW-57/Cx, and J/UW-36/Cx. The Y-axis shows output signal as relative fluorescence units (RFU) from Genebench and the X-axis shows amplicon size (bp). Resulting profile of *Ct* DNA in the presence of commensal/background species (B). Specificity of the 9-plex PCR assay was evaluated against *Neisseria gonorrhoeae (shown), Neisseria flava*, *Neisseria perflava*, *Neisseria lactamica*, *Trichomonas vaginalis, Gardnerella vaginalis*, *Enterococcus faecium*, *Enterococcus faecalis*, *Candida albicans*, and *Candida glabrata*. Amplification reactions were carried out with 50 genome equivalents of *Ct* DNA in the presence of 50,000 genome equivalents of these background DNAs. The 9-plex signature of the *Ct* genomes was unaffected in the presence of the background DNAs; non-specific peaks were readily distinguished from diagnostic amplicons based on molecular weight and attached fluorescent dye.

The article "A Multiplexed Microfluidic PCR Assay for Sensitive and Specific Point-of-Care Detection of Chlamydia trachomatis" was published in 2012. Journal: PLoS One.

### Microfluidic Sanger Sequencing for Discrepant Resolution

PCR amplicons were subjected to microfluidic Sanger sequencing as previously described [23]. Singleplex PCR of the original sample was carried out with similar template DNA amounts and thermal cycling conditions as in the multiplex PCR but using unlabeled primers (Table 1) for both amplification and sequencing. Two microliters from the retrieved PCR products were directly used as template for microfluidic sequencing using the BigDye® Terminator v3.1 cycle sequencing kit (Applied Biosystems, Foster City, CA) and the rapid thermal cycler and microfluidic PCR biochip as described [23]. A total of 18 independent Sanger sequencing reactions (9 forward and 9 reverse) were performed with each reaction containing one sequencing primer (forward or reverse) to obtain bidirectional reads.

**Figure 2:** Representative clinical sample 9-plex profiles. Approximately half the positive electropherograms showed all 9 amplicons with saturated (Panel A) or intermediate (Panel B) peak signals, suggesting high copy numbers of *Ct*. The remaining positive samples generated incomplete profiles, having fewer than 9 amplicons and suggesting low *Ct* numbers. For example, Panel C shows the pCT peak and three other amplicons, Panel D shows pCT and two other amplicons, and Panel E shows no pCT and two other amplicons in blue and red. Panel F is a negative clinical sample showing nonspecific peaks (circled in green) that are readily distinguished from *Ct* amplicons based on molecular weight and fluorescent dye color. The 353 bp peak in blue is readily distinguished from a true 349 bp pCT amplicon in blue. The 230 bp peak in red is readily distinguished from the 4 red-labeled specific amplicons, all of which differ in size from the artifact by at least 120 bp.

### Data Analysis

Samples positive or negative by both multiplex and Amplicor were defined as true positives or true negatives, respectively. For multiplex, samples were called positive when either the pCT locus was present (with or without additional amplicons) or two or more amplicons were present in the absence of pCT. A minimum of two positive amplicons (if the pCT amplicon was not positive) was chosen as a conservative cut off. Discrepant results were resolved by performing PCR on the original sample DNA for all nine loci, and Sanger sequencing the amplicons; discrepants with the correct *Ct* sequence using blastn for at least one locus was considered a true positive. The performance characteristics of multiplex and Amplicor assays for sensitivity, specificity, and positive and negative predictive values were calculated using STATA version 10.0 (StataCorp LP, College Station, TX).

The article "A Multiplexed Microfluidic PCR Assay for Sensitive and Specific Point-of-Care Detection of Chlamydia trachomatis" was published in 2012. Journal: PLoS One.

**Figure 3:** Relative distribution of 68 positive samples with fewer than 9 amplicons observed. Fifty-two samples amplified the pCT (plasmid amplicon) locus; sixteen samples were pCT negative but positive for two or more of the eight remaining loci.

## Results

### Development of the 9-plex Ct Amplification Assay

The multiplex assay was built in three steps: 1) a primer pair for each locus was tested in a singleplex reaction and modified until amplicons were routinely detected in the rapid amplification assay; 2) primer pairs were combined and modified as required until all nine amplicons were routinely detected; and 3) the relative peak heights of the nine loci were balanced such that they were all approximately equal. By design, the peak height of the cryptic plasmid locus was several-fold higher than the rest, reflecting the presence of several cryptic plasmids per *Ct* genome. Figure 1 shows representative profiles of simultaneous amplification of the nine loci in a 20-minute biochip PCR amplification. All nine loci generated amplicons of the expected size.

**Figure 4:** Comparison of multiplex and commercial Amplicor NAAT assays. Prior to discrepant resolution, 129 (49.0%) of 263 of the samples tested were detected positive by the multiplex PCR assay and 94 (35.7%) by Amplicor.

### Evaluation of the Multiplexed Assay on Clinical Samples

The 9-plex microfluidic amplification assay was performed on 263 DNA samples purified from endocervical swabs. To control for run-to-run and lane-to-lane variations in injection efficiency, signal strengths of amplicons were normalized based on the internal size standard marker co-injected with the sample (Average marker signal strength was 3965 RFU with a standard deviation of 2132 RFU.). Resulting electropherograms suggested low, medium, or high numbers of *Ct* genomes per sample based on the number and signal strength of amplicons observed.

**Figure 5:** Sample population distributions of concordant and discordant samples (A) and results of multiplex PCR and Amplicor assays versus sequencing to resolve discordant calls (B). Numbers noted on each bar represent the number of samples that were or were not confirmed by sequencing. Following resolution of discrepants by sequencing, 129 (76+53) and 88 (76+12) samples were positive by multiplex and Amplicor assays, respectively. An overall concordance rate of 82.9% was found between the multiplex assay and sequencing as compared to 17.1% for the Amplicor assay.

The article "A Multiplexed Microfluidic PCR Assay for Sensitive and Specific Point-of-Care Detection of Chlamydia trachomatis" was published in 2012. Journal: PLoS One.

Representative positive electropherograms are illustrated in Figure 2. The 129 positive samples (representing 49% of the swabs tested) ranged from having full profiles containing all nine of the expected amplicons present (61 samples; Figures 2A and 2B) to partial profiles (68 samples; Figures 2C–2E) containing eight or fewer amplicons; 76.5% of these partial profiles contained the pCT amplicon. Figure 3 summarizes the number of amplicons in the partial profiles. Sixteen samples were pCT negative but positive for two or more of the eight remaining loci; 15 of these were Amplicor negative. Nonspecific signals were observed in approximately 20% of electropherograms; these non-specific peaks were readily distinguished from diagnostic amplicons based on molecular weight and attached fluorescent dye (Figure 2F).

### Comparison of Multiplex and Amplicor Assays

Results are presented in Figure 4. Of the 263 samples, 76 were positive and 116 negative by both assays; 129 (76+53 multiplex only) were positive by multiplex and 94 (76, including 8 that were initially Amplicor negative due to inhibitors according to the IC assay but positive on repeat testing, +18 by Amplicor only) by Amplicor. A total of 71 samples were discordant (53 positives by multiplex only and 18 positives by Amplicor only). Of the 71 discrepants, 10 had low DNA amounts and, consequently, less than 20 ng of template was used for the multiplex assay.

### Assessing Discordant Results

To resolve discordant samples, singleplex PCR and Sanger sequencing were performed on the original sample for each of the nine loci. One discordant sample that was negative by multiplex but positive by Amplicor was not sequenced due to insufficient template. It was not possible to sequence Amplicor products directly because the UDP used in the reaction prevents additional post-amplification sequencing.

All 53 samples that were positive by multiplex only were confirmed as positives by sequencing as were the 8 samples with inhibitors by the IC assay. All amplicons generated a sequence with a range of one to nine loci and an average of five loci per sample. Of the 18 samples that were positive by Amplicor only, 12 were confirmed positive (with an average of two loci per sample) and 5 were negative (1 of these 18 samples was not sequenced). All sequenced amplicons gave perfect matches to publicly available whole or partial *Ct* genomes.

The article "A Multiplexed Microfluidic PCR Assay for Sensitive and Specific Point-of-Care Detection of Chlamydia trachomatis" was published in 2012. Journal: PLoS One.

Figure 5 summarizes the sample population distribution and the results of sequencing data for resolving the 71 discrepants. For the multiplex assay, 53 of the 53 positives and 5 of the 17 negatives were confirmed by sequencing. Amplicor showed a much higher error rate with only 12 of the 71 calls confirmed by sequencing (12 of 17 positives, and 0 of 53 negatives not including the indeterminants, which were also confirmed by sequencing).

Based on the above criteria, there were 141 true positives (76 positive by both assays and 65 confirmed by sequencing) and 121 true negatives (116 by both assays and 5 without amplicons for sequencing). The sensitivity and specificity were 91.5% and 100%, and 62.4% and 95.9%, respectively, for multiplex and Amplicor. Moreover, the positive and negative predictive values were 100% and 91% and 94.6% and 68.6%, respectively, for multiplex and Amplicor.

## Discussion

Availability of a rapid, low-cost POC diagnostic for *Ct* would encourage broad screening of both symptomatic and asymptomatic individuals in order to appropriately identify and treat infected patients. Such a test would also likely provide an incentive for the CDC to recommend its use for test-of-cure. Moreover, POC treatment has the potential to reduce the risks associated with *Ct* infections, including HIV-1 infection and transmission, cervical cancer, pelvic inflammatory disease, and infertility [27], [28]. Here, we present data on a diagnostic approach for *Ct* that is rapid and well-suited to adaptation at the POC, and has the potential to be more sensitive and specific than commercial NAATs.

We compared our multiplex assay with the Roche Amplicor NAAT, which targets the cryptic plasmid. Our approach resulted in a higher number of positives [129 (49.0%)] than for Amplicor [88 (33.5%)] following resolution of discrepants by sequencing. Although the number of positives is high, it is unlikely that the amplicons represent DNA from previously treated infection because the samples were from females who had not been on antibiotics in the prior three weeks, and 15 days is limit for detection of DNA in the endocervix following treatment [29]. However, another study showed that DNA can be detected up to 51 days following treatment depending on the NAAT used [30]. Furthermore, the lower numbers for Amplicor are unlikely to be due to DNA degradation as both tests were performed within a similar time frame. However, for the 12 samples that were Amplicor positive and multiplex negative, there may have been insufficient DNA for efficient multiplex amplification, especially since singleplex PCR was able to amplify one to four loci for these 12. Our experiments using 100 ng instead of 20 ng of template for the multiplex reaction for several samples supports this hypothesis.

The article "A Multiplexed Microfluidic PCR Assay for Sensitive and Specific Point-of-Care Detection of Chlamydia trachomatis" was published in 2012. Journal: PLoS One.

The sensitivity of Amplicor for endocervical samples has been reported to range broadly from 64% to 97% [31]–[38]. However, none of these studies sequenced PCR products to resolve discrepants, which may have identified additional true positives. Furthermore, repeat Amplicor testing of the same samples (e.g., positive, negative and equivocal defined as A_450_ absorbance from 0.2 to 0.5) or testing of triplicates of the same sample within the same plate has resulted in vastly different absorbance values ranging from 47.4% to 99.1% [39], [40]. The highest level of agreement was for those with an absorbance of <0.2. Amplicor IC plates were not run in parallel for any of these studies.

The simultaneous interrogation of samples for nine loci increases the probability of detecting *Ct* if there are one or more absent or mutant primer binding sites. This is important, not just because of the problem with detection of many Swedish strains [11], but because of the increasing evidence for recombination and emergence of strains with indels in unpredictable locations [41], [42]. Interestingly, 16 (11.3%) of the 141 true positive samples had no amplicon for the cryptic plasmid, although there were amplicons for 2 to 4 other loci. Fifteen of these were also Amplicor negative. The plasmid has up to 10 copies per organism, which suggests that sufficient DNA should have been available for detection. We are currently examining the molar ratios of the pCT primer sequences to determine if the assay can be further improved.

We found that 11 samples had only one or two amplicon peaks in addition to the cryptic plasmid. The likely explanation would be a low copy number of *Ct* DNA. In such cases, early rounds of amplification may not allow complete binding of all primers, leading to missing peaks. This phenomenon is routinely observed in singleplex amplification reactions, leading to false negatives. Multiplex reactions suffer the same phenomenon [43] but the number of loci present enhance the possibility that one or more loci will be detected successfully.

We identified a high prevalence of *Ct* among our patient population. However, the clinical samples were selected based on known patient risk factors for STDs. Amplicor detected *Ct* in 33.5% of the samples, which is consistent with the known prevalence of *Ct* in our population. Based on our data, we believe that the multiplex approach to *Ct* detection is superior to commercial NAAT detection in that targeting multiple loci allows, in effect, a set of parallel singleplex assays to be performed simultaneously to increase sensitivity and specificity.

The article "A Multiplexed Microfluidic PCR Assay for Sensitive and Specific Point-of-Care Detection of Chlamydia trachomatis" was published in 2012. Journal: PLoS One.

The current multiplex assay can be further improved prior to large-scale clinical trials. For example, the LOD can be enhanced by increasing DNA quantity in the amplification reaction. We have found that 1 µg of genomic DNA is acceptable in our system, which can reduce the number of false negatives (unpublished data). The assay can be further refined by redesigning specific primers to avoid sporadic background hybridization with human DNA. Although this background is readily identified by size and fluorescent label of the peaks (Figure 2), background has the potential to be a larger problem in the presence of much more substrate.

Based on our results, we believe that significant breakthroughs in microfluidic biochip design and fabrication make rapid identification of pathogens in fully-integrated systems a real possibility in the clinical setting. Additional prospective studies will be required in other high risk settings as well as in low to moderate risk settings. Head-to-head comparisons with other NAATs will also be important. We are developing a rapid DNA purification module for urogenital samples that will be integrated with our current amplification, electrophoretic separation, and detection modules into a single ruggedized instrument that can be deployed globally to hospital laboratories, clinics, and field sites as a rapid POC diagnostic for *Ct*.
